RETRACTED

# Dynamic Evaluation of the Rectus Abdominis Muscle before and after Delivery by Ultrasonography

**DOI:** 10.1155/2022/9751136

**Published:** 2022-08-26

**Authors:** Xinxia Wang, Hezhou Li, Bin Luan, Ruizheng Han, Weiwei Lun

**Affiliations:** ^1^Department of Ultrasound, The Third Affiliated Hospital of Zhengzhou University, Zhengzhou, Henan 450052, China; ^2^Department of Pediatrics, The Third Affiliated Hospital of Zhengzhou University, Zhengzhou, Henan 450052, China; ^3^Department of Obstetrics, The Third Affiliated Hospital of Zhengzhou University, Zhengzhou, Henan 450052, China

## Abstract

**Objective:**

To evaluate the changes of rectus abdominis thickness and inter-rectus distance before and after delivery with high-frequency ultrasound.

**Methods:**

A total of 148 pregnant women at 12 weeks of gestation who underwent prenatal examination in our hospital from January 2019 to March 2020 were selected, and 140 of them cooperated with rectus abdominis examination. According to the results of rectus abdominis examination 42 days after delivery, 97 patients were divided into the DRA group with rectus abdominis isolated and 43 patients were divided into the normal group with rectus abdominis not isolated. At 12 weeks, 24 weeks, and 37 weeks of pregnancy, 3 days and 42 days after delivery, the thickness and spacing of the left and right rectus abdominis muscle were measured by high-frequency ultrasound along the white linea at three positions: 5 cm above the navel, 3 cm below the umbilical edge, and 3 cm below the navel.

**Results:**

The thickness of rectus abdominis at 5 cm above the navel, 3 cm below the navel, and at the navel margin of the abdominal white line in the pregnant women of the two groups was gradually decreased with the increase of the pregnancy cycle and gradually recovered after delivery. At 42 days after delivery, the thickness of rectus abdominis in the DRA group was significantly lower than that in the normal group, which was 5 cm above the umbilicus, 3 cm below the umbilicus, and the umbilical margin of the abdominal white line (*P* < 0.05). The space between rectus abdominis 5 cm above the navel, 3 cm below the navel, and the navel margin of the abdominal white line in the pregnant women of the two groups was gradually increased with the increase of the pregnancy cycle and gradually recovered after delivery. At 37 weeks of pregnancy, 3 days after delivery, and 42 days after delivery, the space of rectus abdominis along the umbilicus 5 cm above, 3 cm below the umbilicus, and the umbilicus border of the abdominal white line in the DRA group was significantly larger than that of the normal group (*P* < 0.05).

**Conclusion:**

Ultrasound can accurately measure the inter-rectus distance and rectus thickness, accurately evaluate the degree of DRA, and realize the one-stop evaluation from prenatal diagnosis and prediction to postpartum rehabilitation monitoring, so as to intervene during pregnancy and reduce the risk of postpartum DRA.

RETRACTED

## 1. Introduction

The rectus abdominis of the human body fuses in the midline of the abdomen, and the distance between the rectus abdominis of both sides is no more than 1–2 cm in the normal nonpregnant state. Diastasis recti abdominis (DRA) is caused by acquired factors that cause the separation of the rectus abdominis muscle beyond the normal width along the long axis of the muscle and is characterized by abnormally increased inter-rectus distance, resulting in relaxation and bulging of the abdominal musculature [1–3]. Women are prone to suffering from DRA after delivery. Previous studies have shown that the incidence of DRA is 100%, 60%, 45%, and 32% in the third trimester of pregnancy, 6 weeks, 6 months, and 1 year postpartum, respectively [4, 5]. Generally, DRA is caused by endocrine factors during pregnancy, such as the relaxation of cartilage and ligaments at the joint of sacroiliac joint and phalanx, too much exertion during delivery, and improper posture of the parturient. Without treatment, DRA will not be restored to its normal anatomical position, which can lead to abdominal discomfort and low back pain in the parturient, which will seriously affect women's quality of life [6–8]. Therefore, it is very important to diagnose DRAin time and take early measures to treat it.

At present, the clinical diagnosis of DRA is mainly based on finger-width palpation, but this method has large subjective errors. CT and MRI are also used for DRA diagnosis and evaluation, but the cost is high, and CT has radiation and is not suitable for pregnant women, limiting its clinical application. In recent years, ultrasound has been widely used to detect rectus abdominis and pelvic floor muscles, and its accuracy has been widely recognized [9–11]. In this study, the thickness of rectus abdominis and the distance between rectus abdominis before and after delivery were measured by high-frequency ultrasound, and the changes of rectus abdominis during the whole pregnancy and postpartum period were evaluated, which provided the basis for the diagnosis, prevention, and intervention of DRA.

## 2. Materials and Methods

### 2.1. General Information

A total of 148 pregnant women who underwent prenatal examination and filing in our hospital at 12 weeks of gestation from January 2019 to March 2020 were selected. Of the 148 pregnant women, 140 pregnant women cooperated to complete the rectus abdominis test, 5 pregnant stopped for fetal reasons, and 3 pregnant dropped out of the study. According to the results of rectus abdominis examination 42 days after delivery, 97 patients were divided into the DRA group with rectus abdominis separation and 43 were divided into the normal group without rectus abdominis separation.

RETRACTED

### 2.2. Inclusion Criteria

Singleton and full-term pregnancy; there are no previous reproductive history; there are no complications such as pregnancy-induced hypertension and gestational diabetes mellitus; carry out prenatal examination and delivery in our hospital, and voluntary cooperation with the rectus abdominis examination during pregnancy and postpartum; there is no history of abdominal and pelvic surgery; there is no urinary tract infection during the study.

### 2.3. Exclusion Criteria

Previous history of DRA diagnosis; congenital abdominal wall muscle or nerve defects; previous history of abdominal hernia, urachal fistula, etc.; and inability to lie supine or cooperate with the study due to low back pain.

### 2.4. Method

GE Voluson E8 color Doppler ultrasonic diagnostic apparatus was used with a probe frequency of 7.5 to 12 MHz. Subject level Lie down, place both upper limbs flat on both sides of the body, flex the lower limbs to relax the abdominal muscles, and breathe calmly. The ultrasound probe was placed in the midline of the abdomen, and measurements were made along the white line at three positions: 5 cm above the umbilicus, at the edge of the umbilicus, and 3 cm below the umbilicus along the linea alba. The thickness and spacing of the left and right rectus abdominis were measured by high-frequency ultrasound.

At 12 weeks, 24 weeks, and 37 weeks of pregnancy, 3 days and 42 days after delivery, a high-frequency ultrasound probe was used and was perpendicular to the long axis of the white line and aimed at the distance between the straight muscles on both sides The plane of the probe was perpendicular to the long axis of the rectus abdominis. At the end of each measurement, the still images are collected immediately. The inter-rectus distance is the distance between the hypoechoic medial edges of the rectus abdominis on both sides, the left and right rectus abdominis thickness is the distance between the anterior and posterior fascia of the rectus abdominis, and the maximum diameter is the rectus abdominis thickness. All rectus abdominis examinations were performed by the same attending sonographer, they were measured three times, and an averaged value was taken. Diagnostic criteria of DRA: the lesion site of DRA was divided into infraxiphoid, epigastrium, umbilicus, subumbilicus and above pubic symphysis. DRA was diagnosed when the inter-rectus distance was >20 mm at rest in any part.

RETRACTED

### 2.5. Statistical Methods

SPSS 22.0 software was applied for processing. Age, prepregnancy BMI, postpartum BMI, weight change during pregnancy, abdominal circumference, and other experimental data were expressed by mean ± standard deviation ($\bar{x}$ ± *s*). *T*-test was used to compare the measurement data between groups, and analysis of variance was used to compare multiple groups. The natural birth rate and other counting data are expressed in (%) and compared by pairs *χ*^2^ inspection. The test level is *α* = 0.05, and *P* < 0.05 was considered statistically significant.

## 3. Results

### 3.1. Comparison of General Data of Pregnant and Lying-In Women between the Two Groups

Postpartum BMI, gestational weight change, and abdominal circumference were significantly greater and the rate of spontaneous delivery was significantly lower in the DRA group than in the normal group, and the differences were statistically significant (*P* < 0.05). There was no significant difference in maternal age, prepregnancy BMI, and fetal weight between the two groups (*P* > 0.05), as shown in Table 1.

### 3.2. Ultrasonic Measurement Results of 5 cm Supraumbilical Rectus Abdominis along the Linea Alba in the Two Groups of Pregnant Women

The thickness of the left and right rectus abdominis 5 cm above the umbilicus along the linea alba increased gradually with the pregnancy cycle in both groups. Recovery began postpartum, with left and right rectus muscle thicknesses still lower at 42 days postpartum than at 12 weeks gestation. In the DRA group, there was no significant difference in the thickness of the left and right rectus abdominis 5 cm above the umbilicus along the white line at 12 weeks of pregnancy, 24 weeks of pregnancy, 37 weeks of pregnancy, and 3 days postpartum compared with the normal group (*P* > 0.05). In the DRA group, the thickness of the left and right rectus abdominis 5 cm above the umbilicus along the linea alba at 42 days postpartum was significantly lower than that in the normal group, and the differences were statistically significant (*P* < 0.05).

The rectus abdominis distance of 5 cm above the umbilicus along the linea alba increased gradually with the pregnancy cycle in both the groups. Recovery began postpartum, and the abdominal straight muscle distance was still greater at 42 days postpartum than at 12 weeks of gestation. There was no significant difference in the distance between the rectus abdominis 5 cm above the umbilicus along the linea alba at 12 and 24 weeks of pregnancy between the DRA group and the normal group (*P* > 0.05). The inter-rectus distance of 5 cm above the umbilicus along the linea alba at 37 weeks of gestation, 3 days postpartum, and 42 days postpartum in the DRA group was significantly greater than that in the normal group, and the differences were statistically significant (*P* < 0.05). Figures 1–9.

RETRACTED

### 3.3. Ultrasound Measurements of the Rectus Abdominis 3 cm below the Umbilicus along the Linea Alba in Both Groups

The thickness of the left and right rectus abdominis 3 cm below the umbilicus along the linea alba increased gradually with the pregnancy cycle in both the groups. Recovery began postpartum, with left and right rectus muscle thicknesses still lower at 42 days postpartum than at 12 weeks gestation. In the DRA group, there was no significant difference in the thickness of the left and right rectus abdominis 3 cm below the umbilicus along the linea alba at 12 weeks of pregnancy, 24 weeks of pregnancy, 37 weeks of pregnancy, and 3 days postpartum compared with the normal group (*P* > 0.05). In the DRA group, the thickness of the left and right rectus abdominis 3 cm below the umbilicus along the linea alba at 42 days postpartum was significantly lower than that in the normal group, and the differences were statistically significant (*P* < 0.05).

The rectus abdominis distance 3 cm below the umbilicus along the linea alba increased gradually with the pregnancy cycle in both the groups. Recovery began postpartum, and the abdominal straight muscle distance was still greater at 42 days postpartum than at 12 weeks of gestation. There was no significant difference in the rectus abdominis distance 3 cm below the umbilicus along the linea alba at 12 and 24 weeks of pregnancy between the DRA group and the normal group (*P* > 0.05). The inter-rectus distance 3 cm below the umbilicus along the linea alba at 37 weeks of gestation, 3 days postpartum, and 42 days postpartum in the DRA group was significantly greater than that in the normal group, and the differences were statistically significant (*P* < 0.05).

### 3.4. Ultrasound Measurement Results of Rectus Abdominis at the Umbilical Line of Linea Alba in the Two Groups

The thickness of the left and right rectus abdominis in the umbilical border of the linea alba gradually decreased with the increase of the pregnancy cycle in both the groups. Recovery began postpartum, with left and right rectus muscle thicknesses still lower at 42 days postpartum than at 12 weeks gestation. In the DRA group, there was no significant difference in the thickness of the left and right rectus abdominis of the umbilical border of the linea alba compared with the normal group at 12 weeks of pregnancy, 24 weeks of pregnancy, 37 weeks of pregnancy, and 3 days postpartum (*P* > 0.05). In the DRA group, the thickness of the left and right rectus abdominis in the umbilical border of the linea alba at 42 days postpartum was significantly lower than that in the normal group, and the differences were statistically significant (*P* < 0.05).

RETRACTED

The rectus abdominis interval of umbilical line of linea alba increased gradually with the increase of pregnancy cycle in both the groups. Recovery began postpartum, and the abdominal straight muscle distance was still greater at 42 days postpartum than at 12 weeks of gestation. There was no significant difference in the rectus abdominis distance between the umbilical line of the linea alba at 12 and 24 weeks of gestation in the DRA group and the normal group (*P* > 0.05). In the DRA group, the rectus abdominis intermuscular distance at the umbilical border of the linea alba was significantly greater than that in the normal group at 37 weeks of gestation, 3 days postpartum, and 42 days postpartum, and the differences were statistically significant (*P* < 0.05).

## 4. Discussion

The rectus abdominis is an important muscle structure of the abdominal wall, which is located on both sides of the midline of the anterior abdominal wall, separated by a white line in the middle. Therefore, the position of the abdominal organs will not be affected by the change of gravity and the pressure in the spine, plevis, and abdomen, and assisting normal physiological functions, such as breathing, defecation, and delivery [12, 13]. The inter-rectus distance refers to the width of the linea alba. The linea alba is a reticular fibrous connective tissue extending from the xiphoid process to the pubic symphysis, formed by the intertwining of the external oblique, internal oblique, and trans versus abdominis aponeurosis, which mainly maintains the stability of the abdominal wall and trunk [14, 15]. Clinically, DRA is usually defined by an inter-rectus abdominis distance >2 finger widths. In the management of women during pregnancy and postpartum, DRA is often neglected. With the continuous improvement of medical technology and people's pursuit of healthy life, DRA paid more and more attention to medical workers. The pathogenic factors of DRA are not clear yet, but DRA mostly occurs during pregnancy and postpartum, so it is speculated that its occurrence may be related with pregnancy [16–18].

Ultrasound examination is widely recognized in clinical practice because of its stability, consistency, and reproducibility, and is considered as the gold standard for noninvasive evaluation of DRA. High-resolution probes can directly measure the inter-rectus distance and observe its maximum separation position. Double stitching, virtual wide field of vision, continuous wide field of vision and other imaging are feasible for patients with wide inter-rectus distance in the third trimester [19–21]. Ultrasound wide view imaging technology can generate ultrasound images with a wide field of view, and the key observation area and its surrounding structures can be presented in the same image, which is helpful for the overall understanding and measurement of the image.

RETRACTED

There are also multiple studies on the postpartum rectus abdominis in China, but there are few studies on the postpartum period of the same individual from pregnancy. In this study, we measured the thickness of rectus abdominis and inter-rectus distance before and after delivery by ultrasound to evaluate the changes of rectus abdominis throughout pregnancy and after delivery. It was found that the thickness of rectus abdominis 5 cm above the umbilicus and 3 cm below the umbilicus along the linea alba and at the umbilical line of the linea alba in the two groups decreased gradually with the increase of pregnancy cycle and gradually recovered after delivery. However, the thickness of the rectus abdominis at 42 days postpartum in the DRA group was significantly lower than that in the normal group. With the increase of pregnancy cycle, the inter-rectus distance gradually increases, and it gradually recovered after delivery. At 37 weeks of pregnancy, 3 days postpartum, and 42 days postpartum, there was a significant difference in rectus muscle spacing between the two groups. These results suggest that the inter-rectus distance can directly reflect the situation of DRA, and has an effect on the rectus abdominis at umbilical level. Under the action of estrogen and progesterone, the collagen fibers of pregnant women will gradually expand and stretch, weakening their muscle strength to meet the needs of delivery, while the gradually enlarging fetus and uterus will press pelvic floor muscle tissue and rectus abdominis for a long time, resulting in the damage of muscle tissue, blood vessels, and nerve, and destroying the support system of their abdominal and pelvic organs [22–24]. On the other hand, due to the over extension of the abdominal muscles, the mechanical vector decreases, the position of the white line of the rectus abdominis on both sides is separated, the distance between the rectus abdominis increases abnormally, the strength and support function of abdominal muscle weaken, and other adjacent muscle groups are overloaded, resulting in low back pain, lower stability of the pelvic floor structure, and even displacement of pelvic and abdominal organ in severe cases [25–27].

RETRACTED

This study is a measurement study of DRA from pregnancy to a short time after delivery, which has some limitations. The recovery time of rectus abdominis after delivery is long, and the its influencing factors need further study. At the same time, it is necessary to accumulate cases and conduct large sample, multi-center, and high-quality research.

In summary, ultrasonography can accurately measure inter-rectus distance and rectus thickness, accurately assess the degree of DRA, and achieve a one-stop assessment from prenatal diagnosis prediction to postpartum rehabilitation monitoring for pregnancy intervention.

## Figures and Tables

**Figure 1:** Ultrasound measurement results of the left thickness of the rectus abdominis muscle 5 cm above the umbilicus along the linea alba in both the groups. Note: compared with the normal group, ^*∗*^*P* < 0.05.

**Figure 2:** Ultrasound measurement results of right rectus abdominis muscle thickness 5 cm above the umbilicus along the linea alba in the two groups. Note: compared with the normal group, ^*∗*^*P* < 0.05.

**Figure 3:** Ultrasound measurement results of 5 cm supraumbilical inter-rectus distance along the linea alba in the two groups. Note: compared with the normal group, ^*∗*^*P* < 0.05.

**Figure 4:** Ultrasound measurement results of the left rectus abdominis muscle thickness 3 cm below the umbilicus along the linea alba in the two groups. Note: compared with the normal group, ^*∗*^*P* < 0.05.

**Figure 5:** Ultrasound measurement results of the right rectus abdominis thickness 3 cm below the umbilicus along the linea alba in the two groups. Note: compared with the normal group, ^*∗*^*P* < 0.05.

**Figure 6:** Ultrasound measurement results of the inter-rectus distance 3 cm below the umbilicus along the linea alba in the two groups. Note: compared with the normal group, ^*∗*^*P* < 0.05.

**Figure 7:** Ultrasonographic measurement results of the left rectus abdominis muscle thickness at the umbilical line of linea alba in the two groups. Note: compared with the normal group, ^*∗*^*P* < 0.05.

**Figure 8:** Ultrasonographic measurement results of the right rectus abdominis muscle thickness at the umbilical line of linea alba in the two groups. Note: compared with the normal group, ^*∗*^*P* < 0.05.

**Figure 9:** Ultrasound measurement results of the rectus abdominis intermuscular distance at the umbilical line of linea alba in the two groups. Note: compared with the normal group, ^*∗*^*P* < 0.05.

**Table 1:** Comparison of general data of pregnant and lying-in women in the two groups.

Group	Age (years)	Prepregnancy BMI (kg/m^2^)	Postpartum BMI (kg/m^2^)	Gestational weight change (kg)
Normal group (*n* = 43)	27.93 ± 2.09	20.83 ± 2.71	22.78 ± 2.83	13.87 ± 4.73
DRA group (*n* = 97)	28.16 ± 2.15	20.65 ± 2.59	23.81 ± 2.75	16.89 ± 3.64
*t* value	0.589	0.416	2.026	4.118
*P* value	0.557	0.678	0.045	<0.001

*Group*	*Abdominal circumference (cm)*	*Gestational week (week)*	*Spontaneous delivery*	*Fetal weight (kg)*
Normal group (*n* = 43)	96.56 ± 5.37	38.95 ± 0.53	32	3.16 ± 0.35
DRA group (*n* = 97)	99.70 ± 5.43	39.04 ± 0.69	35	3.22 ± 0.37
*t/χ* ^2^ value	3.167	0.761	17.546	0.899
*P* value	0.002	0.448	<0.001	0.369

RETRACTED

## Data Availability

The data used and/or analyzed during the current study are available from the corresponding author.
